# MicroRNA-346 facilitates cell growth and metastasis, and suppresses cell apoptosis in human non-small cell lung cancer by regulation of XPC/ERK/Snail/E-cadherin pathway

**DOI:** 10.18632/aging.101080

**Published:** 2016-10-18

**Authors:** Cheng-Cao Sun, Shu-Jun Li, Zhan-Peng Yuan, De-Jia Li

**Affiliations:** ^1^ Department of Occupational and Environmental Health, School of Public Health, Wuhan University, 430071 Wuhan, P. R. China; ^2^ Wuhan Hospital for the Prevention and Treatment of Occupational Diseases, 430071 Wuhan, P. R. China; ^3^ Department of Toxicology, School of Public Health, Wuhan University, 430071 Wuhan, P. R. China

**Keywords:** microRNA-346 (miR-346), XPC, non-small cell lung cancer (NSCLC), oncogenesis

## Abstract

Determinants of growth and metastasis in cancer remain of great interest to define. MicroRNAs (miRNAs) have frequently emerged as tumor metastatic regulator by acting on multiple signaling pathways. Here we report the definition of miR-346 as a novel oncogenic microRNA that facilitates non-small cell lung cancer (NSCLC) cell growth and metastasis. XPC, an important DNA damage recognition factor in nucleotide excision repair was defined as a target for down-regulation by miR-346, functioning through direct interaction with the 3′-UTR of XPC mRNA. Blocking miR-346 by an antagomiR was sufficient to inhibit NSCLC cell growth and metastasis, an effect that could be phenol-copied by RNAi-mediated silencing of XPC. In vivo studies established that miR-346 overexpression was sufficient to promote tumor growth by A549 cells in xenografts mice, relative to control cells. Overall, our results defined miR-346 as an oncogenic miRNA in NSCLC, the levels of which contributed to tumor growth and invasive aggressiveness.

## INTRODUCTION

Lung cancer remains a leading cause of cancer-associated mortality worldwide [1–3]. Non-small lung cancer (NSCLC) is responsible for over 80% of lung cancer-related deaths [4]. Despite of great improvements in chemotherapy and molecular-targeted treatment, the survival of this disease remains unsatisfactory. Tumor recurrence and metastasis are frequent and great challenges in the clinical treatment of NSCLC [4]. Thus, identifying novel molecular bio-marker that can inhibit the progression of lung cancer will be urgent for the development of new therapeutic strategies in lung cancer.

Noncoding RNA (ncRNAs) is represented by approximately 97% of transcribed RNA molecules, and only 3% of the RNAs are protein-coding messenger RNAs [5]. MicroRNAs (miRNAs) are a class of small, highly conserved, and non-coding RNAs that directly bind to target genes' 3′-UTRs (3′-untranslated regions) at some sequence-specific sites, which contribute to suppression of these genes expression [6,7]. Increasing evidences have confirmed that ectopic miRNAs are key regulatory factors in various types of cancers [8–12]. Recent studies reveal that miRNAs leads to tumor proliferation, metastasis, apoptosis, stem cell maintenance, cell identity, and senescence [13–18]. Although recent studies on miRNAs have brought mind-blowing insight into our knowledge of human tumors, there are still numerous of unknown details that need to be further elaborated.

MiR-346 (MIMAT0000773), a recognized oncogenic miRNA, has been shown to be played an important role in several diseases. Including Graves' disease [19], rheumatoid arthritis [20], cervical cancer [21,22], cutaneous squamous cell carcinoma [23]. Wang et al. also found that miR-346 regulates osteogenic differen-tiation of human bone marrow-derived mesenchymal stem cells by targeting the Wnt/β-catenin pathway [24]. Moreover, Semaan and his colleagues reported miR-346 controls release of TNF-α protein and stability of its mRNA in rheumatoid arthritis via tristetraprolin stabilization [25]. But up to date, the role of miR-346 on NSCLC has not been investigated yet.

Xeroderma pigmentosum complementation group C (XPC) protein is an important DNA damage recognition factor in nucleotide excision repair [26]. The critical role of XPC in various DNA repair pathways is believed to contribute to the link between the loss of XPC and carcinogenesis of diverse organs [27,28]. In addition to its role in carcinogenesis, XPC deficiency is also associated with a poor prognosis of various cancer patients [27,28]. Mechanistically, XPC deficiency could promote tumor metastatic potential through enhan-cement of matrix metalloproteinase-1 (MMP1) transcription by p53 [29]. Deletion of XPC is associated with early stages of human lung carcinogenesis, and reduced XPC mRNA levels predict poor patient outcome for non-small cell lung cancer (NSCLC) [30]. Recently, Cui and her colleagues revealed that XPC inhibits NSCLC cell proliferation and migration by enhancing E-Cadherin expression [30]. These results suggested that XPC acted as a tumor suppressor in NSCLC.

Our current study is to explore the biological functions of miR-346 in NSCLC and to investigate the underlying mechanisms of its action. We show for the first time that miR-346 directly targets and regulates the full-length 3′-UTR of the human XPC mRNA, which is down-regulated lung cancer. Here, we reported that miR-346 is indeed up-regulated in NSCLC compared with the matching normal lung tissues, and found 3′-UTR of the human XPC mRNA is really a target of miR-346. In conclusion, we reveal that miR-346 facilitates NSCLC cell growth and metastasis in by directly targeting 3′-UTR of XPC.

## RESULTS

### MiR-346 is down-regulated in primary NSCLC tissues and cell lines, and predicts a worse prognosis

miR-346 expression was measured in 114 NSCLC samples and corresponding adjacent normal tissues by qRT-PCR. miR-346 up-regulation was detected in 108/114 (94.74%) of NSCLC tumors (Fig. 1A). Average miR-346 expression was approximately 3.7-fold higher in NSCLC specimens as compared with corresponding adjacent normal tissues (*P* <0.05, Fig. 1A). Next, we examined miR-346 expression in NSCLC cell lines, and results demonstrated a higher expression of miR-346 in A549, SPC-A-1, H1299, 95-D, SK-MES-1, NCI-H520 and NCI-H460 cell lines, compared with that of in normal lung cells 16HBE (Fig. 1B). Although there was no significant association between miR-346 expression and sex, differentiation, or histological tumor type smoking, up-regulated expression of miR-346 was commonly observed in NSCLC patients with elder age, bigger tumor sizes, smokers, positive lymph node metastasis, and advanced stage (*P* <0.05, Table 1). Furthermore, multivariate Cox regression analysis revealed that high (>3.7 folds of increase, n=78) miR-346 expression, elder age, and advanced stage are independent predictors of overall survival in NSCLC patients (Table 2). Kaplan-Meier analysis indicated that high miR-346 expression was associated with poorer overall survival (log-rank test, *P* <0.0001, Fig.1C). Thus, it was concluded that the increased expression of miR-346 might make sense in initiation or development of NSCLC.

**Figure 1:** MiR-346 is up-regulated in primary human lung cancer and NSCLC cell lines, and predicts a worse prognosis

(**A**) miR-346 is significantly increased in primary human lung cancer tissues in comparison to adjacent-normal lung cancer tissues. n=114 for each group. (**B**) The expression level of miR-346 in seven NSCLC cell lines and normal 16HBE cells. Assays were performed in triplicate. (**C**) Kaplan-Meier survival analysis revealed that up-regulated miR-346 is associated with poor prognosis in patients with non-small cell lung cancer. *P < 0.001, Means ± SEM was shown. Statistical analysis was conducted using student t-test.

**Table 1:** Association between miR-346 and baseline characteristics

Parameter	n	miR-346 expression		
		Low(n=38)	High(n=76)	*P*-value[a]
Age(years)				<0.0001[*]
≤ 60	45	26	19	
> 60	69	12	57	
Sex				0.8938
Male	50	17	33	
Female	64	21	43	
Differentiation				0.0873
Well, moderate	36	8	28	
Poor	78	30	48	
Tumor size (maximum diametercm)				0.0061[*]
≤ 3cm	32	18	18	
> 3cm	82	20	62	
Smoking				<0.0001[*]
Yes	83	15	68	
No	31	23	8	
Lymph node metastasis				0.0119[*]
Positive	76	17	59	
Negative	48	21	27	
TMN stage				0.0140[*]
I	21	12	9	
II/III/IV	93	26	67	
Histological tumor type				0.5658
Squamous cell carcinoma	79	25	54	
Adenocarcinoma	35	13	22	

a Chi-square test

* *P*< 0.05

**Table 2:** Influence of miR-346 expression and clinical characteristics on overall survival in NSCLC patients

Factors	Subset	Univariate analysis		Multivariate analysis	
		HR (95%CI)	*P*-value	HR (95%CI)	*P*-value
Age(years)	>60/≤60	2.18 (1.09-2.24)	0.013	1.09 (0.45-0.84)	0.796
Sex	Male/Female	0.94 (0.55-1.70)	0.805		
Differentiation	Poor /Well, moderate	1.26 (0.75-1.66)	0.678		
Tumor size	>3cm/≤3cm	1.78 (0.95-2.48)	0.093		
Smoking	Yes/No	1.60 (0.66-2.33)	0.417		
Lymph node metastasis	Positive/ Negative	2.31 (1.02-3.06)	0.008	2.87 (1.34-5.08)	0.001
TMN stage	(II/III/IV)/I	2.27 (1.23-3.59)	0.003	2.52 (1.14-3.62)	0.002
miR-346	High/Low	6.88 (3.12-8.53)	<0.001	7.645 (3.88-14.30)	<0.001
Histological tumor type	Squamous cell carcinoma/Adenocarcinoma	1.88 (0.86-2.63)	0.717		

HR, hazard ratio; CI, confidence interval.

### Expression of XPC is down-regulated in primary human NSCLC and negatively related to miR-346

XPC is important oncogene that shown strong power of tumorigenesis, by promotion of cell proliferation, metastasis, invasion and epithelial mesenchymal transition (EMT). Thus, we next examined XPC expression in human NSCLC and pair-matched adjacent lung tissues, and our western blot results demonstrated that the expression of XPC protein was significantly decreased in NSCLC tissues compared with lung tissues (Fig. 2A), which were verified by qRT-PCR of XPC mRNA expression (Fig. 2B). Moreover, we evaluated the correlation between XPC mRNA and miR-346 expression in 114 NSCLC tissues, and results revealed expression of XPC mRNA and miR-346 exhibited a significantly inverse correlation as calculated by Pearson correlation (r=−0.51, *P* <0.0001) (Fig. 2C).

**Figure 2:** Expression of *XPC* is up-regulated in primary human lung cancer and negatively expressed related to miR-346 (**A-B**) Western-blot of XPC protein and qRT-PCR of XPC mRNA in lung cancer tissues and adjacent-normal lung cancers. n=114 for each group. **C**. Scatter plots showing the inverse association between miR-346 level and XPC mRNA expression. *P < 0.001, Means ± SEM was shown. Statistical analysis was conducted using student t-test.

### XPC expression is positively correlated with the outcome of NSCLC patients

A previous analysis of 126 NSCLC patients has shown that median survival of patients with lower XPC mRNA levels was shorter compared with patients with higher XPC mRNA levels [34]. To further explore the critical efficiency of XPC in the survival of NSCLC patients, we analyzed the relationship between the XPC mRNA expression level and the survival of NSCLC patients from 2437 lung tumors using publicly available datasets (2015 version) (http://kmplot.com/analysis/index.php?p=service&cancer=lung). The Kaplan-Meier analyses demonstrated that higher XPC mRNA expression in NSCLC patients is correlated with an improvement of the overall survival (OS), as well as progression-free (FP) survival of patients. These correlations are more pro-nounced in patients with adenocarcinoma but not squa-mous cell carcinoma (Fig. 3A–F). These analyses further confirmed the tumor suppressor role of XPC in NSCLC.

**Figure 3:** Prognostic significance of XPC in lung cancer (**A-B**) The effect of XPC mRNA expression level on the overall survival and progression free survival in lung cancer patients was analyzed and the Kaplan-Meier plots were generated by Kaplan-Meier Plotter (http://www.kmplot.com). (**C-D**) The effect of XPC mRNA expression level on the overall survival and progression free survival in lung adenocarcinoma patients was analyzed and the Kaplan-Meier plots were generated by Kaplan-Meier Plotter (http://www.kmplot.com).

### MiR-346 targets human *XPC*

To clarify the relationship between miR-346 and XPC, basic information about hsa-miR-346 was collected from miRBase. XPC is a putative miR-138-5p target predicted by DIANA (Fig. 4A). To verify XPC targeting by miR-346, reporter constructs in which the XPC 3′-UTR, either wild type or mutated in the miR-346 binding sites, was cloned downstream of the luciferase open reading frame (ORF) (Fig. 4A). miR-346 mimic or mimic NC was transfected into A549 and SPC-A-1 cells. When the XPC 3′-UTR was attached to the luciferase gene, luciferase activity decreased significantly (*P* <0.05) in A549 and SPC-A-1 cells transfected with miR-346 mimics, demonstrating that XPC was the target of miR-346 (Fig. 4B). Furthermore, expression of mutant XPC 3′-UTR restored luciferase activity (Fig. 4B). To examine the effect of miR-346 on endogenous XPC expression, we treated A549 and SPC-A-1 cells with NC, miR-346, si-XPC or ASO-346 for indicated time. Western blot assay revealed that both miR-346 and si-XPC treatment decreased the protein level of XPC in A549 and SPC-A-1 cells, while ASO-346 treatment showed an increase in the XPC protein expression than NC treated A549 and SPC-A-1 cells (Fig. 4C).

**Figure 4:** *XPC* proto-oncogene is a target of miR-346 at specific 3′-UTR sites (**A**) The 3′-UTR of *XPC* harbors one miR-346 cognate site. (**B**) Relative luciferase activity of reporter plasmids carrying wild-type or mutant *XPC* 3′-UTR in A549 and SPC-A-1 cells co-transfected with negative control (NC) or miR-346 mimic. (**C**) Protein expression of XPC in A549 and SPC-A-1 cells after transfected with NC, miR-346, si-XPC and ASO-346. Assays were performed in triplicate. *P < 0.001, Means ± SEM was shown. Statistical analysis was conducted using student t-test.

### MiR-346 facilitates cell proliferation and colony formation, and promotes G1/S transition through down-regulation of XPC in NSCLC

miR-346 was ectopically expressed in NSCLC cell lines. We determined the effects of miR-346 over-expression or inhibition, and XPC inhibition on cell proliferation via CCK8 assay. A549 and SPC-A-1 cells (which have high endogenous miR-346 expression) transfected with miR-346 mimics and si-XPC showed increased proliferation (*P* <0.05), which was rescued by ASO-346 treatment (Fig. 5A–B). However, loss of miR-346 suppressed cell proliferation in A549 and SPC-A-1 cells (Fig. 5A–B). To verify these results, we also did the colony formation assay, and results demonstrated miR-346 mimic treatment caused an increase in the clonogenic survival of A549 and SPC-A-1 cells compared with blank A549 and blank SPC-A-1 cells (Fig. 5C), while miR-346 inhibitor-treated A549 cells showed a significant decrease in the clonogenic survival, when compared with blank A549 and blank SPC-A-1 cells (Fig. 5C). Additionally, in A549 and SPC-A-1 cells transfected with miR-346 mimics or si-XPC, the number of cells in G1 phase of the cell cycle decreased and the number in S phase increased (*P* <0.05, Fig. 5C–D), and this was again rescued by ASO-346 treatment (*P*<0.05).

**Figure 5:** The miR-346 affects cell proliferation and cell cycle. A549 and SPC-A-1 cells were analyzed after transfection (**A**-**B**) CCK8 assays of A549 and SPC-A-1 cells after transfected with NC, miR-346, si-XPC and ASO-346. (**C**) Shown are representative photomicrographs of colony formation assay after transfected with NC, miR-346, si-XPC and ASO-346 for fourteen days. (**D-E**) Cell-cycle analysis was performed forty eight hours following the treatment A549 and SPC-A-1 cells with NC, miR-346, si-XPC and ASO-346. The DNA content was quantified by flow cytometric analysis. Assays were performed in triplicate. *P < 0.001, Means ± SEM was shown. Statistical analysis was conducted using student t-test.

### MiR-346 promotes NSCLC cell migration and invasion in vitro

Next, we examined the role of miR-346 on A549 and SPC-A-1 cells migration and invasion. We used Transwell migration approache to assess the role of miR-346 on the ability of A549 and SPC-A-1 cells migration. Results revealed that migration of miR-346 mimic or si-XPC treated cells was increased by 0.32-fold or 0.65-fold in A549 and 0.53-fold or 0.96-fold in SPC-A-1 cells, compared with the blank A549 and SPC-A-1 cells (Fig. 6A–B), respectively. However, when treated with ASO-346, migration in miR-346-expression defected A549 and SPC-A-1 cells were significantly decreased by approximately 48% and 31% relative to blank A549 and SPC-A-1 cells (Fig. 6A–B) respectively.

**Figure 6:** Ectopic expression of miR-346 in A549 and SPC-A-1 cells reduces cell migration and invasion motility (**A-D**) A549 and SPC-A-1 cells were loaded onto the top well of a transwell inserts for cell migration or invasion assay. After twenty four hours, cells that migrated to the bottom chamber containing serum-supplemented medium were stained with 0.1% crystal violet, visualized under a phase-contrast microscope, and photographed. Total number of cells in five fields was counted manually. Assays were performed in triplicate. *P < 0.001, Means ± SEM was shown. Statistical analysis was conducted using student t-test.

To investigate the role of miR-346 on A549 and SPC-A-1 cells invasion, we used a transwell invasion assay. As expected, invasion of miR-346 mimic or si-XPC treated cells was increased by 0.46-fold or 0.54-fold in A549 and 1.1-fold or 0.96-fold in SPC-A-1 cells, relative to the blank A549 and SPC-A-1 cells (Fig. 6C–D), respectively. However, when treated with ASO-346, invasion in miR-346-expression defected A549 and SPC-A-1 cells were significantly decreased by approximately 58% and 49% relative to blank A549 and SPC-A-1 cells (Fig. 6C–D), separately. Taken together, these results clearly demonstrated that miR-346 expression markedly promoted the migration and invasion motility of NSCLC cells through targeting XPC.

### MiR-346 suppresses NSCLC cell apoptosis

We then explored the efficiency of miR-346 on A549 and SPC-A-1 cells apoptosis. Our results of flow cytocytometric analysis revealed that miR-346 mimic or si-XPC treatment contributed to a 62% and 70%, or 56% and 67% of decrease in apoptotic cell death of A549 and SPC-A-1 cells (Fig. 7A–B), respectively. However, the percentage of apoptotic cells induced by miR-346 was increased to the basal level when the cells were treated with the specific miR-346 inhibitor (Fig. 7A–B). In addition, we also tested the caspase-3 and caspase-7 activity after treatment of A549 and SPC-A-1 cells with NC, miR-346 mimic, si-XPC or ASO-346, and results showed that miR-346 mimic and si-XPC treatment significantly decreased the caspase-3 and caspase-7 activity in A549 and SPC-A-1 cell lysate, by approximately 74% and 79%, or 54% and 49% of decrease (caspase-3 activity), 83% and 92%, or 47% and 41% of decrease (caspase-7 activity), than that of in blank A549 and SPC-A-1 cells (Fig. 7C–F), respectively. However, loss of miR-346 by transfecting with ASO-346 remarkably reduced the caspase-3 and caspase-7 activity in A549 and SPC-A-1 cell lysate, compared with that of in blank A549 and blank SPC-A-1 cells (Fig. 7C–F), respectively. These results demonstrated that miR-346 indeed promoted apoptosis in A549 and SPC-A-1 cells.

**Figure 7:** Ectopic expression of miR-346 suppresses apoptosis in A549 and SPC-A-1 cells (**A-B**) Shown are statistical analysis of flow cytometric analysis. (**C-E**) Quantitative representation of caspase-3 and caspase-7 activity in A549 and SPC-A-1 cells transfected with NC, miR-346, si-XPC and ASO-346 for forty eight hours. Assays were performed in triplicate. *P < 0.001, Means ± SEM was shown. Statistical analysis was conducted using student t-test.

### MiR-346 suppresses tumor growth in vivo

To validate the oncogenic role of miR-346 in vivo, we established a BALB/c nude mouse xenograft model using A549 cells. After 8 days, NC, miR-346 mimic, si-XPC or ASO-346 was directly injected into the implanted tumor every 4 days for seven times. The tumor volume was measured every 4 days until day 36. The miR-346 expression was examined by qRT-PCR (Fig. 8C). The tumor volume and weight of mice treated with miR-346 mimic or si-XPC were significantly increased (0.56-fold or 0.38-fold of increase in tumor weight, respectively) relative to that of treated with NC (Fig. 8A–B). While ASO-346 treatment significantly decreased the tumor volume and tumor weight of mice. This result demonstrates miR-346 significantly facilitates the tumorigenicity of A549 cells in the nude mouse xenograft model. In addition, our results of western-blot demonstrated that the decreased expression (48% or 55% of decrease) of XPC in tumors developed from miR-346 mimic or si-XPC treated nude mice relative to that of control tumors (Fig. 8D). Thus, miR-346 promotes the growth of established NSCLC xenografts.

**Figure 8:** Ectopic expression of miR-346 facilitates tumor growth in vivo (**A**) Tumor volume in nude mice. (**B**) Tumor weight in nude mice. Each group contained six mice (n = 6); the data are presented as the mean ± SEM; *p < 0.001, compared with the NC group. (**C**) The expression of miR-346 in nude mice. (**D-F**) The expression of XPC protein in nude mice. Assays were performed in triplicate. *P < 0.001, Means ± SEM are shown. Statistical analysis was conducted using student t-test.

### miR-346 directly targeting XPC and then activating ERK/Snail pathway, which leads to decrease of E-cadherin

It has been reported that the expression of Snail can be down-regulated through the inhibition of the PI3K/AKT or MAPK/ERK pathway [35,36]. And XPC suppressed Snail expression by inhibition of ERK activation [30] (Fig. 9). To investigate whether these pathways are affected by miR-346 modulation, we determined the phosphorylation of ERK1/2 in A549 and SPC-A-1 cells after being transiently transfected with NC, miR-346 mimic, si-XPC or ASO-346.

**Figure 9:** miR-346 directly targeting XPC and then activating ERK/Snail pathway, which leads to decrease of E-cadherin (**A**-**B**) Expression of XPC, phospho-ERK1/2, ERK2, Snail, and E-cadherin were detected in A549 and spc-a-1 cells either transiently transfected with NC, miR-346, si-XPC, or ASO-346. The intensity of XPC, phospho-ERK1/2, ERK2, Snail, and E-cadherin bands were quantified using Image J. Assays were performed in triplicate. *P < 0.05. Means ± SEM was shown. Statistical analysis was conducted using ANOVA.

Results demonstrated both miR-346 mimic and si-XPC suppressed the protein expression of XPC, and then resulted in an increased phosphorylation of ERK1/2 in both A549 and SPC-A-1 cell lines (Fig. 10A–B), indicating that XPC is able to inhibit the ERK pathway in NSCLC cells, and miR-346 could activate ERK pathway by directly targeting XPC. In addition, both miR-346 mimic and XPC knockdown -enhanced Snail expression could be blocked by the inhibition of the ERK pathway, accompanied by an increased expression of E-Cadherin (Fig. 10A–B). These data suggest thatmiR-346 may promote NSCLC cell growth, migration and invasion, and suppress NSCLC cell apoptosis through targeting 3′-UTR of XPC mRNA, leading to inhibition of XPC protein expression, and then contributing to the activation of the ERK pathway. Activated ERK pathway enhances Snail expression, which further suppresses E-Cadherin expression, leading to an accelerated cell proliferation, migration and invasion, and a inhibitory cell apoptosis.

**Figure 10:** Model of the mechanism by which miR-346 suppresses XPC then activating ERK/Snail pathway, which leads to down-regulation of E-Cadherin expression and facilitates cell proliferation and metastasis, and inhibits cell apoptosis in lung cancer. miR-346 directly targeting 3′-UTR of XPC mRNA, contributes to down-regulation of XPC protein. The deficiency of XPC induces the accumulation of the endogenous DNA damage, which activates the ERK pathway. The activated ERK pathway then enhances the expression of Snail, which further represses the expression of E-Cadherin. Decreased expression of E-Cadherin by XPC silencing leads to a promotion of lung cancer cell proliferation and metastasis, and inhibition of lung cancer cell apopt osis.

## DISCUSSION

miRNAs, including oncomiRs or anti-oncomiRs, play crucial roles in the initiation, development and progress-sion of human cancers through post-transcriptional regulation of gene expression [37]. Previous studies indicated that miR-346 might be an oncogenic miRNA in some cancers, including cervical cancer [21,22], cutaneous squamous cell carcinoma [23]. However, the functional role and mechanistic action of miR-346 in NSCLC remained largely unclear. Our study showed miR-346 was upregulated in NSCLC tumor samples as compared with corresponding adjacent normal tissues (Fig. 1). We examined the effects of miR-346 on NSCLC cells in vitro and in vivo.

Our results indicated that miR-346 facilitated NSCLC cell proliferation and promoted the G1/S transition (Fig. 5). In addition, we demonstrated that miR-346 overexpression expedited tumor growth in vivo (Fig. 8). XPC, a DNA repair factor, plays a critical role in preventing carcinogenesis [38,39]. However, the positive correlation between XPC expression and the outcome of various cancer patients including lung, breast, gastric, and ovarian cancer (www.ncbi.nlm.nih.gov) indicates that XPC may play an additional role in preventing tumor progression. It has been reported that XPC deficiency stimulates the invasiveness of lung cancer via inhibition of p27 (kip) and promotion of skp2 and E2F1 [30]. Wu and his colleagues also reported that XPC defects might alter p53 function, which contributing to in the advancement of tumor aggressiveness through increase of MMP1 [40]. In the present study, we provide a novel mechanism for the favorable role of XPC defect in the advancement of NSCLC. Our data reveals that the miR-346-inhibited XPC facilitates the expression of Snail, which further suppresses the expression of E-Cadherin, leading to rescue cancer cells from E-Cadherin-mediated proliferation, migration and invasion inhibition, and apoptosis impetus.

E-Cadherin is frequency low expressed in cancers [41]. E-Cadherin suppressing tumor cell growth and migration in various malignancies is well studied [42]. In the present study, restoration of E-Cadherin expression in miR-346-induced XPC-silencing NSCLC cells can neutralize XPC deficiency-induced cell proliferation, migration and invasion both in vitro and in vivo. Repression of E-Cadherin through E-box-binding pro-teins, such as Snail, Slug, and Zeb1, has been described in many studies [43–45]. Here, we observed an increase of Snail expression at the protein levels and a concomi-tant decrease of E-cadherin expression after miR-346 mimic or si-XPC treatment in lung cancer cell lines.

miRNAs are known to exhibit their biological functions by downregulating expression of their target genes. The predicted miR-346 binding site was present in XPC 3′-UTRs. Whether XPC is the only direct target of miR-346 is still unknown. Luciferase activity assay results verified that XPC was a target of miR-346. XPC levels were decreased by ectopic miR-346 expression in NSCLC cells (Fig. 4). The present study showed that XPC defect in NSCLC cells can rescue them from ASO-346-induced cell cycle arrest and facilitate proliferation (Fig. 5). The oncogenic role of miR-346 in NSCLC is thus at least partly realized by downregulating XPC. Here, we also revealed a direct link between miR-346 and XPC expression in NSCLC patients, and observed that XPC and miR-346 levels were inversely correlated in human NSCLC specimens (Fig. 2C). We also showed that high miR-346 expression correlated with advanced clinical stage and lymph node metastasis. Importantly, high miR-346 (Fig. 1C) and low XPC levels (Fig. 3) were correlated with shorter overall NSCLC patient survival, indicating that miR-346 and XPC may serve as NSCLC biomarkers for clinical outcome prediction, optimal therapy selection and risk group assignment.

In our present study, we discovered that miR-346 and XPC were promising potential prognostic marker for NSCLC, and found miR-346 is dramatically upregulated in human NSCLC tissues compared with normal lung tissues. Moreover, we also revealed up-regulation of miR-346 facilitated NSCLC cell growth, migration and invasion, and promoted G1/S transition, as well as suppressing NSCLC apoptosis through targeting XPC. Our experimental data may provide a strategy that targeting XPC possibly administered by miR-346, might be a clinically effective anti-NSCLC therapeutic strategy.

## MATERIALS AND METHODS

### Tissue collection

Fresh and formalin-fixed, paraffin-embedded, NSCLC tumor tissue samples were obtained from patients who were diagnosed with primary NSCLC. Elective surgery was carried out on these patients at People's Hospital of Wuhan University (Wuhan, China). In total, 20 cases of fresh NSCLC tissues were freshly frozen in liquid nitrogen and stored at −80°C until further use. 114 cases of archived, formalin-fixed, paraffin-embedded NSCLC tissue samples were collected and used in clinic-pathological and prognostic investigation of miR-346. A comprehensive set of clinicopathological data were recorded, including age, gender, size of primary tumor, tumor differentiation, T stage, lymph node metastasis, and distant metastasis. The stage of disease was determined according to the tumor size, lymph node, and metastasis (pTNM) classification system. The use of tissues for this study has been approved by the ethics committee of People's Hospital of Wuhan University. Before using these clinical materials for research purposes, all the patients signed the informed consent. None of these patients received any pre-operative chemotherapy or radiotherapy.

### Cell Culture and transfection

The human NSCLC cell lines, namely, A549, H1299, SPC-A-1, 95D, SK-MES-1, NCI-H520, NCI-H460 and human normal lung epithelial cell line 16HBE were cultured in RPMI-1640 (Invitrogen, Carlsbad, CA, USA) supplemented with 10%. fetal bovine serum (FBS). MiR-346 mimic and mimic negative control, miR-346 inhibitor and inhibitor negative control were purchased from GenePharma Co.,Ltd. (Shanghai, China). Complete medium without antibiotics was used to culture the cells at least twenty-four hours prior to transfection. The cells were washed with 1× PBS (pH7.4) and then transiently transfected with 50 nM NC or miR-346, 100 nM ASO-346 or si-XPC, using Lipofectamine™ 2000 (Invitrogen, Carlsbad, CA, USA) according to the manufacturer's instructions.

### Western blot analysis

Western blot was carried out using the protocol described previously [31–33]. The following primary antibodies were used: rabbit anti-XPC (Santa Cruz, USA), rabbit anti-ERK2 (Santa Cruz, USA), rabbit anti-p-ERK1/2 (Santa Cruz, USA), rabbit anti-Snail (Santa Cruz, USA), anti-E-cadherin (Santa Cruz, USA) and rabbit anti-GAPDH (Santa Cruz, USA).

### RNA isolation and quantitative reverse transcription poly-merase chain reaction (qRT-PCR)

RNA isolation and qRT-PCR was carried out using the protocol described previously [16,17]. GADPH and U6 were used as endogenous controls. In addition, melting curves were used to evaluate non-specific amplification. The relative expression level was calculated using the 2^−ΔΔCt^ method. The primer sequences used in this study are as follows: human XPC: sense: 5′- GACAAGCAGGAGAAGGCAAC-3′, antisense: 5′- GGTTCGGAATCCTCATCAGA-3′; human E-Cadherin: sense: 5′-TGCCCAGAA AATGAA AAAGG-3′, antisense: 5′-GTGTATGTGGCA ATGCGTTC-3′; human Snail: sense: 5′-CCTCAA GATGCACATCCGAAG-3′, antisense: 5′-ACATGGCCTTGTAGCAGCCA-3′; human GAPDH: sense: 5′-GAAGGTGAAGGTCGGAGT-3′, antisense: 5′-GAAGATGGTGATGGGATTTC-3′. The formula and its derivations were obtained from the ABI Prism 7300 sequence detection system user guide. The relative expression values of XPC, E-Cadherin, and Snail were calculated and normalized to GAPDH in each sample and compared. The experiments were performed in triplicates. human GAPDH: sense: 5′-CTCTGCTCCTCCTGTTCGAC-3′, antisense: 5′-ACCAAATCCGTTGACTCCGA -3′.

### Colony formation assay

Colony formation assay was carried out using the protocol described previously [16,17].

### Luciferase Reporter Assays

Luciferase reporter assays was carried out using the protocol described previously [16,17].

### BrdU immunofluorescence assay

BrdU immunofluorescence assay was carried out using the protocol described previously [16,17].

### CCK8 assay

Cell growth was measured using the cell proliferation reagent WST-8 (Roche Biochemicals, Mannheim, Germany). After plating cells in 96-well microtiter plates (Corning Costar, Corning, NY) at 1.0× 10^3^ /well, 10 μL of CCK8 was added to each well at the time of harvest, according to the manufacturer's instructions. One hour after adding CCK8, cellular viability was determined by measuring the absorbance of the converted dye at 450 nm.

### Cell-cycle analysis

Transfected cells were harvested forty-eight hours after transfection. The cells were fixed in 70% ethanol, washed once with PBS, and then labeled with propidium iodide (Sigma-Aldrich) in the presence of RNase A (Sigma-Aldrich) for 30 min in the dark (50 g/mL). Samples were run on a FACSalibur flow cytometer (Becton-Dickinson, FL, NJ, USA), and the percentages of cells within each phase of the cell cycle were analyzed using Cell Quest software.

### Statistical analysis

All experiments were repeated 3 times independently. The results are presented as the means ± standard error mean (SEM). Two independent sample t-test or One-Way Analysis of Variance (ANOVA) was performed using SPSS 19.0 software in order to detect significant differences in measured variables among groups. A value of *P* <0.05 was considered to indicate a statistically significant difference.
